The article "Study on the Effect of Different Endoscopic Auxiliary Treatment of Gastric Mucosal Microtumor" was published in 2022. Journal: Evid Based Complement Alternat Med.

# Study on the Effect of Different Endoscopic Auxiliary Treatment of Gastric Mucosal Microtumor

**DOI:** 10.1155/2022/2557952

**Published:** 2022-10-11

**Authors:** Xiongping Zhong, Fuqun Wang, Dehui Zeng, Yijin Chen, Shengbing Wang

**Affiliations:** Department of Gastroenterology, Meizhou People's Hospital, Meizhou, Guangdong Province, China

## Abstract

**Objective:**

To explore the effect of endoscopy in the treatment of gastric mucosal microtumors.

**Methods:**

A total of 229 patients with gastric mucosal microtumors were treated in our hospital from January 2016 to December 2021. All patients were divided into three groups group A, group B, and group C. Group A was treated with a transparent cap combined with circle-assisted endoscopic resection, group B with ligator combined with circle-assisted endoscopic resection, and group C with endoscopic mucosal tumor resection. The effects of the three groups were observed.

**Results:**

There were 47 patients in group A, 17 males, and 30 females, aged 36–69 years, with an average age of 55.6 ± 9.2 years. There were 54 patients in group B, 18 males, and 36 females, aged 38–72 years, with an average age of 57.6 ± 7.7 years. There were 128 patients in group C, 29 males, and 99 females, aged 33–78 years, with an average age of 55.6 ± 8.4 years. There is no significant difference in age and sex between group A, group B, and group C (*P* > 0.05). The incidence of postoperative complications in group B (66.7%) was significantly higher than that in group A (57.4%) and group C (53.9%) (all *P* < 0.05). The incidence of postoperative complications in group A (57.4%) was higher than that in group C (53.9%), and the difference was statistically significant (*P* < 0.05).

**Conclusion:**

Endoscopic mucosal resection and ligation combined with circle-assisted endoscopic resection are effective and safe in the treatment of gastric mucosal microtumors, but it needs to be combined with targeted nursing measures. The transparent cap combined with ring-assisted endoscopic resection has a significant effect on the treatment of gastric mucosal micromasses, reducing operative complications.

## 1. Introduction

A gastric submucosal tumor is a neoplastic or nonneoplastic space-occupying lesion originating from the tissue below the gastric mucosa [1]. It is a common lesion of the upper digestive tract. On average, 1 case can be found every 200 times of upper gastrointestinal endoscopy [2]. Among them, some small tumors in the gastric mucosa lack clinical symptoms, most of which are found during gastroscopy or other imaging examinations [3]. Patients have only some nonspecific symptoms such as stomach discomfort, nausea, abdominal distension, anorexia, indigestion, and so on [4]. Because of the deep location of the microtumor, it is a difficult problem for clinicians to make an effective treatment plan [5].

The article "Study on the Effect of Different Endoscopic Auxiliary Treatment of Gastric Mucosal Microtumor" was published in 2022. Journal: Evid Based Complement Alternat Med.

In recent years, with the improvement of people's health awareness and living standards, endoscopic technology has been rapidly developed and widely used, and the level of diagnosis and treatment has been gradually improved [6]. A variety of endoscopic resection techniques have been used in the diagnosis and treatment of gastric submucosal tumors [7]. Compared with surgery, endoscopic resection has the advantages of a definite curative effect, high safety, less trauma, and quick recovery [8]. At present, the existing endoscopic treatment techniques include transparent cap combined with circle-assisted endoscopic resection, ligator combined with circle-assisted endoscopic resection, endoscopic mucosal tumor resection, and so on [9]. Endoscopic mucosal tumor resection has a better surgical effect and less risk, so it has been used as a standard measure for endoscopic treatment of gastric mucosal microtumors [10]. At the same time, other endoscopic resection based on this technique has also been gradually developed and applied in the clinic, such as transparent cap combined with circle-assisted endoscopic resection and ligator combined with circle-assisted endoscopic resection, which is used in the clinic [11]. Gastric submucosal tumors are a safe and effective treatment, with the advantages of simple operation and less trauma, reduce patient mortality, and improve patients' quality of life, which has been promoted and applied in the clinic [12].

At present, there are many studies on gastric submucosal masses, but there are still some deficiencies in the domestic and foreign studies on the efficacy of endoscopic-assisted treatment of gastric mucosal micromasses at home and abroad [13]. The application of endoscopic-assisted treatment of gastric mucosal micromasses is still controversial [14]. In summary, it is particularly important to pay attention to the endoscopic treatment of gastric mucosal microtumors [15]. This study retrospectively studied the clinical data of patients who had been treated under endoscopy and had identified the pathological type as gastric mucosal microtumors in our hospital, explored the application efficacy of different ways of endoscopic-assisted treatment of gastric mucosal microtumors, and analyzed the clinical effects of different endoscopic treatment, so as to provide more reference basis for clinical workers in the endoscopic diagnosis and treatment of gastric mucosal microtumors.

## 2. Methods

### 2.1. Study Design and Participants

A total of 229 patients with gastric mucosal microtumors from January 2016 to December 2021 were selected. All patients were randomly divided into three groups: group A, group B, and group C. There were 47 patients in group A, 17 males, and 30 females, aged 36–69 years. There were 54 patients in group B, 18 males, and 36 females, aged 38–72 years. There were 128 patients in group C, 29 males, and 99 females, aged 33–78 years. All subjects obtained informed consent. The ethics committee of Meizhou People's Hospital approved the research plan. All participants underwent a complete medical history and clinical examination.

The article "Study on the Effect of Different Endoscopic Auxiliary Treatment of Gastric Mucosal Microtumor" was published in 2022. Journal: Evid Based Complement Alternat Med.

### 2.2. Inclusion and Exclusion Criteria

Inclusion criteria were as follows: (1) Patients who met the diagnostic criteria of gastric submucosal tumors in the guidelines for Clinical diagnosis and treatment of tumors and were diagnosed by imaging examination. (2) Patients and their families knew about the study, the purpose of examination, and the possible risks of the operation, agreed to endoscopic treatment or surgical treatment, and signed the informed consent form. (3) Smooth gastric mucosa without ulcer, no lymph node, and distant metastasis. (4) Complete postoperative follow-up data. Exclusion criteria were as follows: (1) Patients with digestive tract stricture and perforation. (2) Patients with acute inflammation of the digestive tract. (3) Patients with heart, lung, brain, kidney, and other important organ failure or dysfunction, and who could not tolerate anesthesia. (4) Those who take anticoagulants, hematological diseases, and blood coagulation disorders.

### 2.3. Observation Index

The comparison of postoperative complications was as follows:

Postoperative patients fasted with water, were routinely treated with acid suppression, nutritional support, and mucosal repair and were observed for complications such as dyspnea, fever, hematemesis, gastrointestinal bleeding, or abdominal distension.

From the date of discharge, the patients were followed up by telephone, WeChat, and other means. The patients were asked to return to the clinic for gastroscopy or ultrasonic gastroscopy for 3∼6 months and 1 year to observe and evaluate the wound healing status and whether there were complications such as residual lesions or recurrence.

### 2.4. Statistical Analysis

The SPSS23.0 statistical software was used to process the data, in which (*x* ± *s*) represented the measurement data, while the counting data were expressed by the number of cases (*n*), (%) represented the intergroup rate, and the comparison between groups was made by the analysis of variance. The difference was statistically significant (*P* < 0.05).

## 3. Result

A total of 229 patients with gastric mucosal microtumors from January 2016 to June 2021 were selected. All patients were randomly divided into three groups group A, group B, and group C. There were 47 patients in group A, 17 males, and 30 females, aged 36–69 years, with an average age of 55.6 ± 9.2 years. There were 54 patients in group B, 18 males, and 36 females, aged 38–72 years, with an average age of 57.6 ± 7.7 years. There were 128 patients in group C, 29 males, and 99 females, aged 33–78 years, with an average age of 55.6 ± 8.4 years. There was no difference in the age, sex, intraoperative blood loss, intraoperative perforation rate, and endoscopic complete resection rate of the selected patients (*P* > 0.05), Table 1.

The article "Study on the Effect of Different Endoscopic Auxiliary Treatment of Gastric Mucosal Microtumor" was published in 2022. Journal: Evid Based Complement Alternat Med.

### 3.1. Comparison of Complication Rates among the Three Groups

The incidence of postoperative complications in group B was significantly higher than that in group A and group C (all *P* < 0.05). The incidence of postoperative complications in group A was higher than that in group C, and the difference was statistically significant (*P* < 0.05), Table 2.

## 4. Discussion

A gastric submucosal tumor is one of the most common clinical tumors [16]. In recent years, although the incidence of gastric submucosal tumors is increasing year by year, the overall prognosis of the disease is good. Surgery or endoscopic resection is the main treatment [17, 18]. The gastric submucosal tumor is a kind of lesion that originated from the submucous layer, its surface is covered by normal mucosal tissue, showing as a protuberant lesion, and routine biopsy usually cannot obtain an accurate pathological diagnosis, so it has a high risk of malignant transformation [19, 20]. The main clinical manifestations are gastrointestinal obstruction, gastrointestinal bleeding, abdominal pain, and fever, which seriously threaten the life safety and quality of life of patients [21].

Conventional laparotomy is the most important and effective treatment for large gastric submucosal tumors [22]. Endoscopic treatment is mainly used for patients with small submucosal tumors (< 20 mm), of which endoscopic submucosal tumor resection is more effective and less risky for submucosal tumors with diameters of 10–20 mm, endoscopic mucosal resection is a minimally invasive procedure for the treatment of submucosal tumors of the gastrointestinal tract, the utility model has the advantages of accurate positioning, high block resection rate, reducing the chance of residual and recurrence, realizing radical treatment, less trauma, few complications, no change of the structure of the digestive tract, safety and effectiveness in treating the pathological changes of the digestive tract and so on [23, 24]. At present, it has been accepted by international endoscopists and is widely used in the endoscopic resection of digestive tract lesions [25]. Now it has been used as a standard measure for endoscopic treatment of submucosal gastric masses. However, for gastric submucosal tumors with smaller diameters (< 10 mm), endoscopic mucosal resection is too complex and difficult to operate [26–28]. Therefore, transparent cap-assisted endoscopic full-thickness resection is also known as transparent cap suction tumor stripping, which is gradually applied in the clinic. Transparent cap-assisted endoscopic full-thickness resection has the advantages of simple and fast operation, short operation time, high resection integrity rate, and sufficient postoperative resection tissue for the identification of the nature of gastric submucosal tumors with a diameter of less than 10 mm [29].

The article "Study on the Effect of Different Endoscopic Auxiliary Treatment of Gastric Mucosal Microtumor" was published in 2022. Journal: Evid Based Complement Alternat Med.

The results of this study showed that the incidence of complications in group A was lower than those in group B. The results show that a transparent cap combined with ring-assisted endoscopic resection is very beneficial to the treatment of gastric mucosal microtumors, reducing the incidence of complications. The results show that a transparent cap combined with ring-assisted endoscopic resection can effectively promote early postoperative recovery and reduce the incidence of complications.

Based on the above findings, although endoscopic mucosal resection and ligator combined with circle-assisted endoscopic resection with ligator combined with ligation are effective and safe measures for the treatment of gastric mucosal microtumors, they should also be combined with targeted nursing measures. In order to reduce the amount of intraoperative bleeding and reduce the incidence of complications. The transparent cap combined with ring-assisted endoscopic resection has a significant effect on the treatment of small gastric mucosal tumors, reduces surgical complications, and improves the level of diagnosis and treatment. In conclusion, the transparent cap combined with ring-assisted endoscopic resection is more suitable for the endoscopic treatment of small gastric mucosal tumors.

## Figures and Tables

**Table 1:** Baseline characteristics of participants.

	Group A (*N* = 47)	Group B (*N* = 54)	Group C (*N* = 128)
Gender (male/female, example)	17/30	18/36	29/99
Age (*x* ± *S*, year)	55.6 ± 9.2	57.6 ± 7.7	55.6 ± 8.4
Intraoperative blood loss (ml)	0.2 ± 0.9	0.3 ± 1.2	3.1 ± 10.0
Intraoperative perforation rate (%)	82.1%	83.3%	40.8%
Endoscopic complete resection rate (%)	93.6%	92.8%	92.5%

**Table 2:** Comparison of the incidence of complications among the three groups (*n* (%)).

Group	*n*	Dyspnea	Fever	Abdominal distension	Gastrointestinal bleeding	Abdominal pain	Total incidence (%)
Group A	47	0 (0)	2 (4.3)	1 (2.1)	0 (0)	24 (51.1)	27 (57.4)
Group B	54	0 (0)	1 (1.9)	5 (9.3)	0 (0)	30 (55.6)	36 (66.7)
Group C	128	0 (0)	3 (2.3)	4 (3.1)	2 (1.6)	60 (46.9)	69 (53.9)

The article "Study on the Effect of Different Endoscopic Auxiliary Treatment of Gastric Mucosal Microtumor" was published in 2022. Journal: Evid Based Complement Alternat Med.

## Data Availability

The data used to support the findings of this study are available from the corresponding author upon request.
